# Multimodal Imaging of Target Detection Algorithm under Artificial Intelligence in the Diagnosis of Early Breast Cancer

**DOI:** 10.1155/2022/9322937

**Published:** 2022-01-10

**Authors:** Meiping Jiang, Sanlin Lei, Junhui Zhang, Liqiong Hou, Meixiang Zhang, Yingchun Luo

**Affiliations:** ^1^Department of Ultrasonography, Hunan Province Maternal and Child Health Care Hospital, Changsha 410008, Hunan, China; ^2^Department of Surgery, The Second Xiangya Hospital, Central South University, Changsha 410011, Hunan, China; ^3^NHC Key Laboratory of Birth Defect for Research and Prevention (Hunan Provincial Maternal and Child Health Care Hospital), Changsha 410100, Hunan, China

## Abstract

This study aimed to analyze the diagnostic value of multimodal images based on artificial intelligence target detection algorithms for early breast cancer, so as to provide help for clinical imaging examinations of breast cancer. This article combined residual block with inception block, constructed a new target detection algorithm to detect breast lumps, used deep convolutional neural network and ultrasound imaging in diagnosing benign and malignant breast lumps, took breast density grading with mammography, compared the convolutional neural network (CNN) algorithm with the proposed algorithm, and then applied the proposed algorithm to the diagnosis of 120 female patients with breast lumps. According to the results, accuracy rates of breast lump detection (94.76%), benign and malignant breast lumps diagnosis (98.22%), and breast grading (93.65%) with the algorithm applied in this study were significantly higher than those (75.67%, 87.23%, and 79.54%) with CNN algorithm, and the difference was statistically significant (*P* < 0.05); among 62 patients with malignant breast lumps of the 120 patients with breast lumps, 37 were patients with invasive ductal carcinoma, 8 with lobular carcinoma in situ, 16 with intraductal carcinoma, and 4 with mucinous carcinoma; among the remaining 58 patients with benign breast lumps, 28 were patients with fibrocystic breast disease, 17 with intraductal papilloma, 4 with breast hyperplasia, and 9 with adenopathy; the differences in shape, growth direction, edge, and internal echo of multimodal ultrasound imaging of patients with benign and malignant breast lumps had statistical significance (*P* < 0.05); the malignant constituent ratios of patients with breast density grades I to IV were 0%, 7.10%, 80.40%, and 100%, respectively. In short, the multimodal imaging diagnosis under the algorithm in this article was superior to CNN algorithm in all aspects; according to the judgment on benign and malignant breast lumps and breast density with multimodal imaging features, the higher the breast density, the higher the probability of breast cancer.

## 1. Introduction

Breast cancer is a malignant tumor with the highest incidence among women [1]. According to incomplete statistics, the number of new patients of breast cancer in our country takes a percentage of 12.5% in the total number of patients in the world each year, and the mortality rate takes a percentage of 9.7% in the global mortality rate [2]. According to study, the high incidence of breast cancer is in the 70–80 year-olds in developed countries, while this brings forward for 20 years in our country [3]. Moreover, for the differences in regions and medical levels in our country, people's understanding on breast cancer is not deep enough in relatively backward areas, which often results in advanced breast cancer when discovered [4]. Therefore, early and accurate diagnosis and treatment of the early breast cancer have become a key in improving the cure rate [5]. In addition to breast biopsy, imaging examination has become a common and important method for medical diagnosis of breast cancer, including ultrasound (US), computer tomography (CT), mammography, magnetic resonance imaging (MRI), and three-dimensional digital breast tomography (DBT) [6,7]. Multimodal imaging technology is an emerging technology in recent years. It combines multiple imaging technologies and fusing information from different modal images to obtain multiple aspects of the body at the same time, so that information complementation and cross-validation are possible. The biological detection system based on multimodal images can provide more comprehensive physiological and pathological information for the research of life and medical science and provide a quantitative detection and evaluation platform for the development of advanced diagnosis and treatment methods [8].

With the development of artificial intelligence and information technology, neural network has been applied in medical images [9]. Elastography ultrasound imaging technology can be used to evaluate the hardness of biological soft tissues, and change of the hardness may indicate the lump [10]. Pan et al. [11] use grid-based algorithm to segment breast lumps automatically, extract elastic features from elastic ultrasound images, and analyze benign and malignant lumps with the features of B-mode ultrasound. Breast density is of vital importance in the diagnosis of breast cancer. For individual difference of radiology staff and addition of supervisory factors, there are many problems with breast density grading, thus the grading accuracy needs to be improved [12]. Kirschnick et al. [13] propose an 8-layer convolutional neural network (CNN), which extracts the imaging features of mammogram images, achieves a good breast density grading, and divides the tissues into dense and adipose tissues. Although numerous scientific researchers have been committed to the studies on benign and malignant breast lumps diagnosis and breast density grading, most of the studies are single-imaging studies [14].

In this study, 120 female patients with breast lumps who were admitted to our hospital from July 4, 2017, to July 5, 2020, were selected as the research samples, and all of them underwent multimodal imaging examinations. Then, based on the residual block and Google's Inception module, an artificial intelligence target detection algorithm was proposed and applied to analyze the multimodal images of patients. In addition, the imaging characteristics of patients' benign and malignant lesions were analyzed to comprehensively evaluate the value of multimodal imaging based on artificial intelligence target detection algorithms for early diagnosis of breast cancer.

## 2. Materials and Methods

### 2.1. Research Objects

120 female patients aged 20–76 years with breast lumps in hospital from July 4, 2017, to July 5, 2020, were selected as research subjects. This study had been approved by the Ethics Committee of the hospital, and the patients and their families had understood this study and signed the informed consent form.

The inclusion criteria were defined as follows: patients with breast lumps less than 20 mm in diameter; patients not receiving chemotherapy, surgery, or medication before surgery; patients accepted multimodal imaging examinations before surgery; patients with case results after biopsy.

The exclusion criteria were determined as follows: patients not signing the informed consent; patients with incomplete clinical data; patients withdrawn from experiment midway due to personal reasons; patients in pregnancy and lactation.

### 2.2. Multimodal Image Examination

Multimodal ultrasound examination used color Doppler ultrasound diagnostic equipment, which was equipped with elastic imaging software Toshiba Aplio500/400, and the probe frequency was 6–13 MHz. Before the examination, patient was kept in a supine position under the guidance of medical staff, with arms raised to ensure the exposure of breasts and axillas, and then gray-scale ultrasound was used to give cross-sectional scan. During the period, it needs to observe distribution, size, and growth environment of the lesions, as well as their connection with surroundings, etc. Finally, by switching to the elastography mode, two-dimensional ultrasound image and the corresponding ultrasound elastography image could be observed via the real-time display function, and adjustment should be given according to the specific situation to obtain elastic ultrasound image.

Mammography adopted MammoNovation Siemens FFDM with amorphous selenium solid-state detector, pixel size 60 mm (micrometers), 14-bit contrast resolution, and 3328 × 4084 pixels in matrix, to save the image acquired.

### 2.3. Multimodal Imaging of Target Detection Algorithm under Artificial Intelligence

#### 2.3.1. Breast Lump Detection with the Ultrasonic Images under Target Detection Algorithm

The target detection algorithm was mainly divided into two-stage target detector and single-stage target detector: the former had high accuracy rate and took a long time for the interest area extraction specially, and the latter had low accuracy rate and a fast-running speed. According to the lumps and the characteristics of real-time ultrasound imaging, single-stage target detector was used to improve accuracy of breast lump detection by improving the network and optimizing the loss function. SSD model was constructed in this article by combining residual block with Google's inception block. Deep CNN was affected by many factors, and small blocks were reused in this article. Residual blocks of different network scales are shown in Figure 1.

SSD is single-stage detector algorithm. It firstly draws forward features and reverse optimization from CNN, extracts interest areas, and then performs nonmaximum suppression to obtain the final prediction results. By setting *k* frames in a certain position, targeting category *c*, and confirming each frame with 4 offset values, the number of convolution kernels *K* needed is as below:

(1) $$\begin{array}{c} K=\left(c+4\right)\times k. \end{array}$$

The number of results in the extracted feature map *m* × *n* is as below:

(2) $$\begin{array}{c} N=\left(c+4\right)\times k\times m\times n. \end{array}$$

The frame label of original image corresponds to the object border in the feature map, and the default box is matched with any groundtruth box (a). In this article, jaccard overlap (b) between the two was selected to be greater than the threshold 0.5, and intersection ratio of the two can be expressed as below:

(3) $$\begin{array}{c} j\left(a,b\right)=\frac{\left|a\cap b\right|}{\left|a\cup b\right|}=\frac{\left|a\cap b\right|}{\left|a\right|+\left|b\right|-\left|a\cap b\right|}, \end{array}$$

*y*_*ij*_^*q*^=1 is used to indicate that *a* in series *i* matches with *b* phase in series *j* in category *q*, and *y*_*ij*_^*q*^=0 does not match. According to the matching strategy in this article, it must be *y*_*ij*_^*q*^ ≥ 1. Total objective loss function can be expressed as below:

(4) $$\begin{array}{c} F\left(X,C,L,G\right)=\frac{\left[L_{\text{conf}}\left(X,C\right)+\lambda L_{\mathrm{loc}}\left(X,L,G\right)\right]}{n}. \end{array}$$

In (4), *n* refers to the number of matches between the two, *loc* refers to the input localization loss; conf refers to confidence loss, which is loss function of Softmax. Improvement was given to Softmax in this article. Binary grading is taken as an example, and cross entropy *H* is expressed as below:

(5) $$\begin{array}{c} H\left(P,Y\right)=\left\{\begin{array}{cc} -\log\left(P\right), & Y=1,\\ -\log\left(1-P\right), & \mathrm{otherwise}, \end{array}\right) \end{array}$$

(6) $$\begin{array}{c} P_{T}=\left\{\begin{array}{cc} P, & Y=1,\\ 1-P, & \mathrm{otherwise}. \end{array}\right) \end{array}$$

The equation below can be obtained by combining (5) and (6):

(7) $$\begin{array}{c} H\left(P,Y\right)=H\left(P_{T}\right)=-\log\left(P_{T}\right). \end{array}$$

After improving cross entropy and adding coefficient *β*_*T*_, the definition is as below:

(8) $$\begin{array}{c} \beta_{T}=\left\{\begin{array}{cc} \beta , & \mathrm{label}=1,\\ 1-\beta , & \mathrm{label}=-1, \end{array}\right)\left(0\leq \beta \leq 1\right). \end{array}$$

By taking (8) in (7), it can be obtained in

(9) $$\begin{array}{c} H\left(P_{T}\right)=-\beta_{T}\log\left(P_{T}\right). \end{array}$$

The deeper the number of layers of many CNNs, the smaller the resolution of characteristics patterns. When giving prediction with *n* characteristics patterns, the size *S*_*K*_ of each characteristics pattern can be expressed as

(10) $$\begin{array}{c} S_{K}=S_{\min}+\frac{\left(S_{\max}-S_{\min}\right)\left(K-1\right)}{n-1},K\in \left[1,n\right]. \end{array}$$

In (10), scale of the highest level *S*_max_=0.93 and that of the lowest level *S*_min_=0.30 are taken. When expressing with *β*_*r*_, it is as below:

(11) $$\begin{array}{c} \beta_{r}=\left(1,2,3,\frac{1}{2},\frac{1}{3}\right). \end{array}$$

The width and height of each default frame can be calculated with

(12) $$\begin{array}{c} W_{K}^{\beta }=S_{K}\sqrt{\beta_{r}}, \end{array}$$

(13) $$\begin{array}{c} H_{K}^{\beta }=\frac{S_{K}}{\sqrt{\beta_{r}}}. \end{array}$$

When the ratio of width to height of the default frame is 1, one default frame is added, and there are total 6 frames in each feature map. Algorithm flow is shown in Figure 2.

#### 2.3.2. Benign and Malignant Breast Lumps Diagnosis with Elastic Ultrasound Images under CNN

After obtaining interest areas, it needs to subtract B-mode ultrasound images from the elastic ultrasound images to obtain pure elastic information, which is then converted into H channel images. The conversion process is as below:

(14) $$\begin{array}{c} H=\;\cos^{-1}\left[\frac{0.5\left[\left(r-g\right)+\left(r-b\right)\right]}{\sqrt{{\left(r-b\right)}^{2}+\left(r-b\right)\left(g-b\right)}}\right]. \end{array}$$

In (14), ranges of the red, green, and blue values of the pixels in images *r*, *g*, and *b* are in 0–360. In this article, data was augmented by data enhancement to prevent overfitting, including image selection, translation, and flipping. The automatic feature extraction was realized before image training. The convolution operation is expressed as below:

(15) $$\begin{array}{c} E_{l+1}=\delta_{l+1}\left(W_{l+1}\times E_{l}+b_{l+1}\right)l+1. \end{array}$$

In (15), *l* and *l*+1 refer to previous and current layers; *b* and *W* refer to bias and weight; *E* is output; and *δ* is activation function. After convolution, the maximum pooling and depooling shall occur:

(16) $$\begin{array}{c} E_{l,\mathrm{pooling}}=\max\mathrm{pooling}\left(E_{l}\right). \end{array}$$

The network of lumps grading is in the following layers, and the nonlinear activation function Softmax is expressed as below:

(17) $$\begin{array}{c} E_{l}=\mathrm{softmax}\left(W_{l}\times E_{l-1}+b_{l}\right),\\ \mathrm{softmax}=\frac{e^{a_{i}}}{\sum e^{a_{i}}}. \end{array}$$

The subsequent process of CNN is deconvolution, which is used to update weights and biases, and seeks the optimum parameters by optimizing the multiclass cross entropy loss function.

(18) $$\begin{array}{c} p=E\left(\tau ,X\right). \end{array}$$

In (18), *τ* refers to all weights and biases and *X* refers to input. Algorithm flow is shown in Figure 3.

#### 2.3.3. Breast Density Grading with Mammography under CNN

The thinking of breast density grading under CNN is consistent with that of benign and malignant breast lumps diagnosis. This article just added residual block in the deep CNN to extract deeper features for the convenience of breast density grading. Algorithm flow is shown in Figure 4.

### 2.4. Simulation Experiment

  I. Breast lump detection with the ultrasonic image of target detection algorithm: workstation was dell-7910, two E5-2640v4 Intel Haswells CPUs were configured, the optimization algorithm was Adam, the maximum number of iterations was 10,000, the initial learning rate was 0.0001, weight was initialized randomly, and bias was initialized to 0.
  II. Diagnosis of benign and malignant breast lumps with elastic ultrasound images under CNN: experimental framework was Keras, Tensorboard was used to monitor network training, workstation was dell-7910, two E5-2640v4 Intel Haswells CPUs were configured, the optimization algorithm was Adam, Batch size was 8, the maximum number of iterations was 6,000, and the initial learning rate was 0.0001.
  III. Breast density grading by mammography under CNN: experimental framework was Keras, Tensorboard was used to monitor network training, workstation was dell-7910, two E5-2640v4 Intel Haswells CPUs were configured, the optimization algorithm was Adam, Batch size was 8, the maximum number of iterations was 3,000, the initial learning rate was 0.0001, weight was initialized randomly, and bias was initialized to 0.

### 2.5. Performance Evaluation Indicators

Accuracy rates of the two algorithms in breast lump detection were compared, and intersection and union ratio (IoU) was used to evaluate the overlap between target area *A* and actual label *B*. When IoU > 0.75, lump detection was considered to be correct, and the accuracy rate should be calculated:

(19) $$\begin{array}{c} \text{IoU}=\frac{\left|A\cap B\right|}{\left|A\cup B\right|}. \end{array}$$

The two algorithms were compared in the sensitivity, specificity, and accuracy rate of benign and malignant breast lumps diagnosis:

(20) $$\begin{array}{c} \mathrm{sensitivity}=\frac{\mathrm{TP}}{\mathrm{TP+FN}}\times \mathrm{100\%,} \end{array}$$

(21) $$\begin{array}{c} \mathrm{specificity}=\frac{\mathrm{TN}}{\mathrm{TN+FP}}\times \mathrm{100\%,} \end{array}$$

(22) $$\begin{array}{c} \mathrm{accuracy}\;\mathrm{rate}=\frac{\mathrm{TP+TN}}{\mathrm{Total}}\times \mathrm{100\%}. \end{array}$$

In (20), (21), and (22), *TP* refers to correct identification of malignant lumps; *TN* refers to correct identification of benign lumps; *FP* refers to incorrect identification of malignant lumps; *FN* refers to incorrect identification of benign masses.

Accuracy rates of the two algorithms in breast density grading were compared. Breast density can be divided into four grades. Grade I is fat type with very low density (0%–25%); Grade II is scattered glandular type with low density (26%–50%); Grade III is uneven dense type with relatively high and uneven density (51%–75%); Grade IV is dense type with extremely high density (76%–100%).

Pathological results and multimodal ultrasound imaging features (shape, growth direction, edge, and internal echo) of benign and malignant lesions of the patients were recorded, and malignant constituent ratio of breast density grading of the patients was calculated:

(23) $$\begin{array}{c} \mathrm{constituent}\;\mathrm{ratio=}\frac{\mathrm{malignant}\;\mathrm{number}}{\mathrm{graded}\;\mathrm{number}\;\mathrm{of}\;\mathrm{people}}\mathrm{\times 100\%}. \end{array}$$

### 2.6. Statistical Method

The data processing of this study adopted SPSS 22.0 version statistical software, the measurement data was expressed as mean value ± standard deviation (‾*x* ± *s*), the counting data was expressed in percentage (%), and the difference was statistically significant at *P* < 0.05.

## 3. Results

### 3.1. Pathological Results of All Patients

Figures 5 and 6 gave pathological results of malignant and benign lumps, respectively. The figure illustrated that there were 62 patients with malignant breast lumps in the 120 patients with breast lumps, including 37 patients with invasive ductal carcinoma, 8 with lobular carcinoma in situ, 16 with intraductal carcinoma, and 4 with mucinous carcinoma, and that there are 58 patients with benign breast lumps, including 28 patients with fibrocystic breast disease, 17 with intraductal papilloma, 4 with breast hyperplasia, and 9 with adenopathy.

### 3.2. Comparison of Accuracy Rates of the Two Algorithms in Breast Lump Detection

Figure 7 showed the comparison of accuracy rates of the two algorithms in breast ump detection.  Figure 6 was a schematic diagram of breast lump detection under the algorithm proposed in this study, where *IoU* > 0.75. The figure indicated that the accuracy rate of breast lump detection under CNN algorithm was 75.67%, and that under the algorithm proposed in this study was 94.76%. The accuracy rate of breast lump detection under the algorithm proposed in this study was significantly higher than that under CNN algorithm, and the difference was statistically significant (*P* < 0.05).(Figure 8)

### 3.3. Comparison of the Two Algorithms in Benign and Malignant Breast Lump Detection

Figure 9 shows comparison of the two algorithms in benign and malignant breast lump detection. The figure indicated that the sensitivity of benign and malignant breast lump detection under CNN algorithm was 84.23%, the specificity was 82.74%, and the accuracy rate was 87.23%; the sensitivity of benign and malignant breast lump detection under the algorithm proposed in this study was 97.13%, the specificity was 94.32%, and the accuracy rate was 98.22%. The sensitivity, specificity, and accuracy rate of benign and malignant breast lump detection under the algorithm proposed in this study were significantly higher than those under CNN algorithm, and the differences all had statistical significance (*P* < 0.05).  Figure 10 shows the ultrasound images of different breast masses. The first column was ultrasound images of benign masses, and the second and third columns were ultrasound images of malignant masses. The darker the color (red), the harder the mass and the more severe the lesion.

### 3.4. Comparison of Accuracy Rates of the Two Algorithms in Breast Density Grading

Figure 11 showed comparison of accuracy rates of the two algorithms in breast density grading.  Figure 12 revealed that the accuracy rates of Grades I, II, III, and IV and the overall accuracy rates under CNN algorithm were 77.8%, 85.65%, 83.45%, 68.00%, and 79.54%, respectively, and those under the algorithm proposed in this study were 97.89%, 96.23%, 96.45%, 87.54%, and 93.65%, respectively. The accuracy rate of breast density grading under the algorithm proposed in this study was significantly higher than that under CNN algorithm, and the differences were all significant statistically (*P* < 0.05).

Figure 12 shows mammograms of different breast density grades. Grade I was fat type; Grade II was scattered glandular type; Grade III was uneven dense type; Grade IV was dense type.

### 3.5. Comparison of Multimodal Ultrasound Image Features of Patients with Benign and Malignant Breast Lumps

Figure 13 gave comparison of multimodal ultrasound image features of patients with benign and malignant breast lumps. The figure illustrated that 65.5% (38/58) of benign lumps had regular shape, and 34.5% (20/58) had irregular shape, 70.7% (41/58) showed parallel growth direction, and 29.3% (17/58) showed nonparallel growth direction, 56.9% (33/58) had complete edges, and 43.1% (25/58) had incomplete edges, 20.7% (12/58) gave even internal echo, and 79.3% (46/58) gave uneven internal echo; and that 22.6% (14/58) of malignant lumps had regular shape, and 77.4% (48/58) had irregular shape, 95.2% (59/58) showed parallel growth direction, and 4.8% (3/58) showed nonparallel growth direction, 25.8% (16/58) had complete edges, and 74.2% (46/58) had incomplete edges, 71.0% (44/58) gave even internal echo, and 29.0% (18/58) gave uneven internal echo. The differences in shape, growth direction, edge, and internal echo of multimodal ultrasound images of patients with benign and malignant breast lumps were significant statistically (*P* < 0.05).

### 3.6. Malignant Constituent Ratio of Breast Density Grades of Patients

Figure 14 indicated malignant constituent ratio of breast density grades of patients. The figure illustrated that there were 4, 28, 56, and 32 patients in breast density Grades I, II, III, and IV, respectively, and that malignant constituent ratios were 0%, 7.10%, 80.40%, and 100%, respectively, which revealed the higher the breast density grade, the higher the probability of malignant lumps.

## 4. Discussion

At present, breast cancer has become a major disabling and fatal disease among middle-aged and elderly women worldwide, greatly affecting the physical and mental health of women. Vigorously publicizing the early detection, early diagnosis, and early prevention of breast cancer can effectively improve the 5-year survival rate of patients and effectively reduce the economic burden on the family and society of patients with breast disease [15–17]. Multimodal ultrasound imaging technology has broad application prospects in the field of breast cancer diagnosis. It can conduct multiparameter and all-round evaluations for early breast cancer patients and subsequent neoadjuvant chemotherapy, and better guide clinical evaluation and prognosis improvement [18]. As inspired by multimodal imaging omics, this article combined residual block with inception block, constructed a new target detection algorithm to detect breast lumps, used deep CNN and ultrasound imaging in diagnosing benign and malignant breast lumps, took breast density grading with mammography, and gave comparison with CNN algorithm. The results revealed that the accuracy rate of breast lump detection under the algorithm proposed in this study (94.76%) was significantly higher than that under CNN algorithm (75.67%), and the difference was statistically significant (*P* < 0.05). The sensitivity (97.13%), specificity (94.32%), and accuracy rate (98.22%) of benign and malignant breast lump detection under the algorithm proposed in this study were significantly higher than those under CNN algorithm (84.23%, 82.74%, and 87.23%), and the differences had statistical significance (*P* < 0.05). The accuracy rate of breast density grading under the algorithm proposed in this study (93.65%) was significantly higher than that under CNN algorithm (79.54%), and the differences were significant statistically (*P* < 0.05). This indicated that the multimodal imaging of target detection algorithm under artificial intelligence proposed in this article could improve the accuracy rates of breast lump detection, benign and malignant breast lumps diagnosis, and breast grading. Such results were similar to the study results of Yoo et al. [19]. The combination of multimodal imaging and deep CNN realizes breast lumps diagnosis and breast density grading and indicates a higher accuracy rate by comparing with traditional diagnostic methods.

Later, it was applied to the diagnosis of 120 female patients with breast lumps, and the results showed that there were 62 patients with malignant breast lumps, including 37 patients with invasive ductal carcinoma, 8 with lobular carcinoma in situ, 16 with intraductal carcinoma, and 4 with mucinous carcinoma, and that there were 58 patients with benign breast lumps, including 28 patients with fibrocystic breast disease, 17 with intraductal papilloma, 4 with breast hyperplasia, and 9 with adenopathy. 65.5% (38/58) of benign lumps had regular shape, and 34.5% (20/58) had irregular shape, 70.7% (41/58) showed parallel growth direction, and 29.3% (17/58) showed nonparallel growth direction, 56.9% (33/58) had complete edges, and 43.1% (25/58) had incomplete edges, 20.7% (12/58) gave even internal echo, and 79.3% (46/58) gave uneven internal echo; 22.6% (14/58) of malignant lumps had regular shape, and 77.4% (48/58) had irregular shape, 95.2% (59/58) showed parallel growth direction, and 4.8% (3/58) showed non-parallel, 25.8% (16/58) had complete edges, and 74.2% (46/58) had incomplete edges, 71.0% (44/58) gave even internal echo, and 29.0% (18/58) gave uneven internal echo. The differences in shape, growth direction, edge, and internal echo of multimodal ultrasound images of patients with benign and malignant breast lumps were significant statistically (*P* < 0.05). This was consistent with the study results of Ulaner (2019) [20], who applied the FDG PET/CT to the initial stage of breast cancer, treatment response assessment, and suspected recurrence assessment, and compared it with other imaging methods; it was found that FDG PET/CT was currently the imaging method that had the greatest impact on the clinical management of breast cancer patients. Ultrasound elastography could clearly identify the boundaries of breast lumps and provide growth information of the lumps; thereby the judgment on benign and malignant lumps might be given with image features. There were 4, 28, 56, and 32 patients in breast density Grades I, II, III, and IV, respectively, and malignant constituent ratios were 0%, 7.10%, 80.40%, and 100%, respectively. This identifies with the study results of Skaane et al. (2019) [21] and indicates that the risk of breast cancer of patients in dense breast type is about 5 times higher than that in nondense breast type, and the higher the breast density, the higher the risk of breast cancer [22].

## 5. Conclusion

Inspired by multimodal imaging omics, this article combined residual block with inception block, constructed a new target detection algorithm to detect breast lumps, used deep CNN and ultrasound imaging in diagnosing benign and malignant breast lumps, took breast density grading with mammography, and gave comparison with CNN algorithm. Later, it was applied to the diagnosis of 120 female patients with breast lumps. The results indicated that multimodal imaging of target detection algorithm under artificial intelligence could improve the accuracy rates of breast lump detection, benign and malignant breast lumps diagnosis, and breast grading; the higher the breast density, the higher the incidence of breast cancer, according to the judgment on benign and malignant breast lumps and the density with multimodal imaging features. However, the sample size of patients selected in this study was small with simple source, and the results may be biased. Follow-up studies should further expand the inclusion of patient samples and conduct multicenter and large-scale discussions. All in all, the results of this article provided theoretical support for the early diagnosis and treatment of breast cancer.

## Figures and Tables

**Figure 1:** Residual blocks of different network scales: (a) original block, (b) bottleneck block, and (c) inception block.

**Figure 2:** Algorithm flow.

**Figure 3:** Algorithm flow.

**Figure 4:** Algorithm flow.

**Figure 5:** Pathological results of malignant lumps.

**Figure 6:** Pathological results of benign lumps.

**Figure 7:** Comparison of accuracy rates of the two algorithms in breast ump detection. *Note.* ∗ indicated that the difference compared to CNN algorithm was statistically significant ((*P* < 0.05).

**Figure 8:** Schematic diagram of breast lump detection under this detection.

**Figure 9:** Comparison of the two algorithms in benign and malignant breast lump detection. *Note.* ∗ indicated that the differences compared to CNN algorithm had statistical significance ((*P* < 0.05).

**Figure 10:** Comparison of ultrasound images of benign and malignant breast lumps. *Note.* A_1_ ∼ C_1_ were elastic ultrasound images; *A*_2_ ∼ C_2_ were B-mode ultrasound images; A_1_ and *A*_2_ show benign lumps; B_1_, B_2_, C_1_, and C_2_ show the malignant lumps.

**Figure 11:** Comparison of accuracy rates of the two algorithms in breast density grading. *Note.* ∗ indicated that the differences compared to CNN algorithm were significant statistically (*P* < 0.05).

**Figure 12:** Mammograms of different breast density grades: (a) Grade (I), (b) Grade II, (c) Grade III, and (d) Grade IV.

**Figure 13:** Comparison of multimodal ultrasound image features of patients with benign and malignant breast lumps. *Note.* ∗ revealed that the differences compared to benign lumps were significant statistically (*P* < 0.05).

**Figure 14:** Malignant constituent ratio of breast density grades of patients.

## Data Availability

The data used to support the findings of this study are available from the corresponding author upon request.
